# Predicting the Herd Immunity Threshold during an Outbreak: A Recursive Approach

**DOI:** 10.1371/journal.pone.0004168

**Published:** 2009-01-09

**Authors:** Nathan T. Georgette

**Affiliations:** Science Department, Allen D. Nease High School, Ponte Vedra, Florida, United States of America; University of Bern, Switzerland

## Abstract

**Background:**

The objective was to develop a novel algorithm that can predict, based on field survey data, the minimum vaccination coverage required to reduce the mean number of infections per infectious individual to less than one (the Outbreak Response Immunization Threshold or ORIT) from up to six days in the advance.

**Methodology/Principal Findings:**

First, the relationship between the rate of immunization and the ORIT was analyzed to establish a link. This relationship served as the basis for the development of a recursive algorithm that predicts the ORIT using survey data from two consecutive days. The algorithm was tested using data from two actual measles outbreaks. The prediction day difference (PDD) was defined as the number of days between the second day of data input and the day of the prediction. The effects of different PDDs on the prediction error were analyzed, and it was found that a PDD of 5 minimized the error in the prediction. In addition, I developed a model demonstrating the relationship between changes in the vaccination coverage and changes in the individual reproduction number.

**Conclusions/Significance:**

The predictive algorithm for the ORIT generates a viable prediction of the minimum number of vaccines required to stop an outbreak in real time. With this knowledge, the outbreak control agency may plan to expend the lowest amount of funds required stop an outbreak, allowing the diversion of the funds saved to other areas of medical need.

## Introduction

The World Health Organization (WHO) has emphasized case management over outbreak response immunization (ORI) based on cost-effectiveness per mortality avoided [1], [2], demonstrating that cost is a significant issue with regard to ORI. However, studies have demonstrated the effectiveness of ORI at limiting the spread of a VPD and thus reducing the number of resulting morbidities and mortalities [1]–[3].

Vaccination has two purposes: 1) individual protection, and 2) population or “herd” protection [4]. This research focuses on determining the minimum number of vaccines required to achieve the population protection. In other words, the objective is to predict the minimum vaccination coverage required to reduce the mean number of secondary infections per infectious individual to less than unity. Poorer nations may choose to focus on achieving population protection rather than on ensuring individual protection for as many as possible to conserve funds in resource poor settings. The method proposed in this paper demonstrates a manner through which impoverished countries may predict the number of vaccines necessary to achieve protection of the population and thus preserve funds.

### Key Definitions

As two terms with similar meanings are used throughout this paper, I will clarify the distinctions:

- Herd Immunity Threshold: The overall fraction of a population that must be vaccinated (regardless of when these vaccinations occur) to reduce the mean number of secondary infections per infectious individual to less than one for a VPD [5]. This threshold level reduces the probability of infection of unimmunized persons, thus essentially granting indirect protection to those without immunity and thereby gradually stopping the outbreak [5]. An alternative definition has been offered [6], which would characterize the above approach as “herd effect” rather than the herd immunity threshold. The noun “threshold” is used to reflect the quantitative nature of the phenomenon. Herd Immunity Threshold = Pre-Outbreak Vaccine Coverage+ORIT.
- Outbreak Response Immunization Threshold (ORIT): The fraction of a population that must be vaccinated during the outbreak to reduce the mean number of secondary infections per infectious individual to less than one, thus causing the cessation of the outbreak. It should be noted that achieving the ORIT also results in the achievement of the herd immunity threshold.

By attaining the ORIT, the outbreak control agency may reduce the probability of infection among the unimmunized to a sufficient degree, thus gradually stopping the outbreak [5]. The ORIT may be guaranteed, at a rather high financial cost, by immunizing as much of the population as possible. This high expenditure is problematic since measles, along with most VPDs, primarily affects the poorest nations around the world [7]. In addition, implementing an ORI program of the scale required to end an outbreak requires a large expenditure of resources in the form of vaccines and personnel [8]. Therefore, immunizing the minimum number of persons required to achieve the ORIT can preserve critical resources in a poor nation. These resources may be diverted to other areas of dire medical concern. By immunizing only the minimum number of persons required to gradually stop an outbreak the outbreak control agency can save vaccines for a later date. For example, unused MMR vaccines, with an average shelf life of 2 years according to the Centers for Disease Control and Prevention [9], may be employed at a later date to help stop a future outbreak.

To immunize the minimum number of persons to stop an outbreak, the outbreak control agency must have advance knowledge of an approximation for the ORIT. This prediction would also grant an outbreak control agency several days to prepare, plan for, and coordinate a massive immunization drive according to this target value, thus improving the overall efficiency of outbreak control.

### Other approaches

The herd immunity threshold is most often presented as being dependent on the mean number of infections caused by a single infectious individual during his/her duration of infectiousness [10], [11], which is defined as the individual reproduction number [12] in this paper. Several time-based models for a variety of reproduction numbers have been developed previously, with some recent examples including [9], [12]–[15], through which the individual reproduction number (synonymous with the effective reproduction number), and by extension the ORIT, may be predicted. With the individual reproduction number, the ORIT may be approximated by solving for the vaccination coverage that satisfies *R_i_*<1 where *R_i_* is the individual reproduction number [4]. In other words, when the ORIT is achieved, each infectious person infects less than one other person on average, resulting in the ending of an outbreak [5].

Other methods for determining the minimum vaccination deployment required to end an outbreak have been developed. One notable perspective involves the “firefighter problem,” first introduced in [16], in which the minimum number of firefighters required to control a fire spreading through a grid is calculated. In the epidemiological application of this problem, the fire is a VPD and the firefighters are vaccines, protecting the vertices at which they are located. In other words, the minimum number of vaccines needed to contain the outbreak may be solved for through an iterative algorithm solution to the firefighter problem. Significant advances have been made on this front, including the examination of grids with three or more dimensions [17], and even generalization for grids of several dimensions [18].

### Purpose

This paper proposes a simple and readily applicable recursive predictive algorithm based on a tractable model I previously developed (hereinafter the “Threshold Model”) for the ORIT in [19]. This research builds on that previous work. The outbreak control agency may use this predictive algorithm to obtain an accurate prediction of the ORIT from up to six days in advance based on survey data input from two prior days. The paper then goes on to analyze the effects of a variety of factors on the accuracy of the prediction. In addition, I develop a novel formulation for determining the effects of additional vaccination on changes in the individual reproduction number.

## Methods

### Underlying model

The Threshold Model proposed earlier [19] is as follows:(1)In the Threshold Model, *P* is the initial fraction of a population susceptible, *I* is the fraction of the population infectious, *R* is the fraction of a population recovered,  is the recovery rate (fraction of the infectious persons that recover per day), *S* is the fraction of a population susceptible, *N* is the initial fraction of the population infectious, and  is the immunization rate, where the value for  may be calculated with the following equation: (2)In (1), the *V_T_* term is the most critical aspect. It represents the fraction of the population that must be immunized during the outbreak to achieve the herd immunity threshold, and is defined as the Outbreak Response Immunization Threshold (ORIT) in this paper. As most populations have high pre-outbreak immunity rates (often around 0.80 [20], [21]), the actual herd immunity threshold is calculated as: Pre-Outbreak Immunization Coverage+*V_T_*. Thus, *V_T_* values in this paper will be significantly lower than the largely accepted value of the herd immunity threshold for measles, which is around 0.90 [1].

In many cases, a significant portion of the population has been immunized during the outbreak before the ORIT is calculated using the Threshold Model in (1). The Threshold Model calculates the total fraction of the population that must be immunized during the outbreak to achieve the herd immunity threshold, not the fraction remaining. In other words, the fraction of the population that must be immunized from the point of calculation onwards is equal to: ORIT–fraction already immunized during the outbreak.

In addition, (1) is based on a system of differential equations (which itself is based on the classic SIR model) that assumes homogenous mixing of the population and the mass action principle [19]. It also does not incorporate household mixing, outbreak response protocols (except vaccination), or the fraction of the population exposed but not infectious [19]. While these assumptions limit the accuracy of the Threshold Model, they simultaneously allow for greater simplicity and real time applicability.

Based on the planned recursive nature of the predictive algorithm and the lack of data available for its testing (the number of infections and immunizations per day) a specific plan is established. The first stage, development, includes the analysis of the 2003 Republic of Marshall Islands (RMI) measles outbreak [20]. The second stage, testing, includes the application of the predictive algorithm to the 2003 RMI outbreak (also used in development) and a new test data set for the 2006 Fiji measles outbreak [21]. Data from both the 2003 RMI outbreak [20] and the 2006 Fiji measles outbreak [21] also was used to test the Threshold Model [19].

### Development of ORIT algorithm

To develop the recursive predictive algorithm, I first graph the Threshold Model's estimations for the ORIT over the duration of the 2003 Republic of Marshall Islands (RMI) measles outbreak [20]. Measles is chosen due to its high impact on poor nations and its high infectiousness [7]. This graph is presented in **Figure 1**.

**Figure 1:** To begin to understand the trends in the changes in the Outbreak Response Immunization Threshold (ORIT), I calculate the ORIT, using the Threshold Model, at several points during the 2003 RMI measles outbreak. I also graph the fraction of the population immunized during the outbreak.

A strong relationship between the changes in the ORIT and the rate of immunization is noticeable. With this in mind, I posit the following inverse, direct, and constant relationships:(3.1)
(3.2)
(3.3)Where *k* is an arbitrary constant of proportionality and *t* is time, in days. As ρ is a fraction, the 4th root is taken to increase its magnitude. This higher value reflects the high impact of ρ on changes in the ORIT.

I first calculate the change in the ORIT between two consecutive days for several instances during the 2003 RMI measles outbreak and find significant variation in this slope among the tested instances. This variability in the slope of the ORIT line (an approximation for ) eliminates the possibility that  is constant, thus eliminating (3.3). A comparison of the slopes at each of these points with their respective immunization rates () demonstrates that the slope and immunization rate are close to inversely proportional. I conclude that the inverse relationship (3.1) is the most reasonable possibility and find that (3.1) only applies when .

To generate a recursive model based on this function, the value of *k* must constantly update in a recursive fashion. Based on this necessity, I apply a modified form of Euler's method with secant, rather than tangent, lines. First, the slope of the secant line (defined as *m*) over the two previous days is found to be:(4)With (4), the value for *k* may be calculated based on the relationship between *m* and  in the following equation: (5)I set  as an approximation for  based on the previous constant of proportionality calculated in (5). The definition of  is shown below:(6)Therefore, the basic recursive formula for the value of  is generated as follows based on the modified version of Euler's method discussed above: (7)Inserting (4) into (5), then (5) into (6), and finally (6) into (7) yields the final recursive definition with which the ORIT may be predicted: (8)The final recursive definition described in (8) predicts *V_T_* several days in advance by first predicting *V_T_* for the very next day. Using this prediction, the threshold for the following day is predicted and this procedure is repeated until the final value is determined.

To expedite the application of the recursive predictor, I develop an algorithm for the prediction of the ORIT using the recursive formula in (8) for the Java programming language, which I call the Recursive Prediction of the ORIT Algorithm (RPORITA).

The application of the RPORITA consists of the following steps:

1. Enter the background information of the outbreak, including total population, vaccination coverage at beginning of outbreak, and recovery rate (defined as 1/8 for measles [7] in this paper).
2. Enter the survey data for two consecutive days, including number of persons infectious and recovered for each day and total number of persons immunized during the outbreak for each day.
3. Select the day number for which the herd immunity threshold should be predicted and enter the number of immunizations that will occur on each day until the day of prediction.
4. The RPORITA then returns the predicted ORIT for the selected day of prediction.

### Development of an individual reproduction number model

The ability to determine the effects of additional vaccination on the individual reproduction number would provide insight into outbreak response and improving cost effectiveness. For this reason, I seek to develop a model for , the change in the individual reproduction number, as a function of , the change in the vaccination coverage. To approximate this relationship, I solve for *dR_i_*/*dV*.

The model for the individual reproduction number I developed concurrently with the Threshold Model in [19] is as follows: (9)By introducing variables into equation (2) from above, the formulation for the immunization rate becomes: (10)With *V* = the fraction of the population immunized during the outbreak, *c* = the current day number, and *b* = the day number on which vaccination began during the outbreak. The vaccinations that cause the  are assumed to occur instantaneously for the purposes of this model. Therefore, both *c* and *I* are held constant. However, *S* would decrease due to the increase in *V* caused by the vaccinations, yielding the relationship below: (11)To simplify the *R_i_* function, I decompose it into functions of its numerator and denominator, or *y* and *z*, respectively. (12)
(13)Taking the derivatives of the numerator and denominator individually with respect to *V* yields: (14)
(15)By the quotient rule for differentiation: (16)Inserting (12,13,14,15) into (16) results in: (17)To determine the effects of changes in *V* on *R_i_* at extremely low incremental values, the following approximation is established:(18)By (18),  can be determined with the function below:(19)


## Results

### Measles outbreak application

I predict the ORIT for an approximate 20 day period with an average of 5 day intervals for both datasets [20], [21]. The interval of the highest rate of immunization was chosen for the test period. The numerical results of these applications are presented in **Tables 1** **and** **2**, and the graphical depictions can be seen in **Figure 2**.

**Figure 2:** This figure presents a graphical depiction of the comparison between the Recursive Prediction of the Outbreak Response Immunization Threshold Algorithm (RPORITA) prediction for the Outbreak Response Immunization Threshold (ORIT) and the Threshold Model estimation based on direct data input. I apply the RPORITA to both the 2006 Fiji measles outbreak (A) and the 2003 RMI measles outbreak (B). I show the RPORITA prediction generated with each prediction day difference (PDD).

**Table 1:** Comparison of the RPORITA-generated predictions for the ORIT and ORIT approximations based on direct input of survey data for the 2006 Fiji measles outbreak.

Date (DSI)	Threshold Model estimated ORIT	RPORITA prediction average	Prediction error based on average	RPORITA predicted ORIT	Prediction error	PDD
3/29 (9)	0.1528	0.1454	−0.0074	0.1469	−0.0059	4
				0.1452	−0.0076	5
				0.1440	−0.0088	6
4/03 (14)	0.1326	0.1329	−0.0003	0.1330	0.0004	4
				0.1358	0.0032	5
				0.1299	−0.0027	6
4/08 (19)	0.1135	0.1122	−0.0013	0.1131	−0.0004	4
				0.1113	−0.0022	5
				0.1122	−0.0013	6
4/14 (25)	0.1045	0.1027	−0.0018	0.0969	−0.0076	4
				0.1081	0.0036	5
				0.1032	−0.0013	6
4/18 (29)	0.0919	0.0926	0.0007	0.0975	0.0056	4
				0.0956	0.0037	5
				0.0846	−0.0073	6

The RPORITA signifies the Recursive Prediction of the Outbreak Response Immunization Threshold Algorithm, which I use to produce a comparison of the RPORITA prediction and the Threshold Model approximation for the ORIT, or Outbreak Response Immunization Threshold, based on direct data input. The prediction day difference (PDD) is the difference between the second day of direct input on which the prediction is based and the day of the prediction. The Days since Start of Immunization (DSI) is the number of days between the day of prediction and the start of the ORI. The prediction error is defined as follows: prediction error = RPORITA prediction−Threshold Model approximation.

**Table 2:** Comparison of RPORITA-generated predictions for the ORIT and ORIT approximations based on direct input of survey data for the 2003 RMI measles outbreak.

Date (DSI)	Threshold Model estimated ORIT	RPORITA prediction average	Prediction error based on average	RPORITA predicted ORIT	Prediction error	PDD
8/20 (19)	0.1292	0.1319	0.0027	0.1348	0.0056	4
				0.1300	0.0008	5
				0.1308	0.0016	6
8/25 (24)	0.1212	0.1200	−0.0012	0.1158	−0.0054	4
				0.1169	−0.0043	5
				0.1272	0.0060	6
8/30 (29)	0.1166	0.1182	0.0016	0.1156	−0.0010	4
				0.1198	0.0032	5
				0.1192	0.0026	6
9/05 (35)	0.1074	0.1106	0.0032	0.1090	0.0016	4
				0.1105	0.0031	5
				0.1123	0.0049	6
9/10 (40)	0.1016	0.0995	0.0021	0.0992	−0.0024	4
				0.0993	−0.0023	5
				0.0999	−0.0017	6

The RPORITA signifies the Recursive Prediction of the Outbreak Response Immunization Threshold Algorithm, which I use to produce a comparison of the RPORITA prediction and the Threshold Model approximation for the ORIT, or Outbreak Response Immunization Threshold based on direct data input. The prediction day difference (PDD) is the difference between the second day of direct input on which the prediction is based and the day of the prediction. The Days since Start of Immunization (DSI) is the number of days between the day of prediction and the start of the ORI. The prediction error is defined as follows: prediction error = RPORITA prediction−Threshold Model approximation.

### Error Analysis

The number of days between the second day of direct data input and the day of the prediction can be defined as the Prediction Day Difference (PDD). I define the difference between the day of prediction and the beginning of ORI as Days since Start of Immunization (DSI). To better understand the specific factors affecting the level of prediction error of the RPORITA, two relationships were examined: 1) between DSI and prediction error, and 2) between PDD and prediction error. These relationships are examined using data from both outbreaks, allowing several conclusions to be drawn.

**Tables 1** **and** **2** illustrate several key aspects of the RPORITA. First, all of the prediction errors are within 0.009 of the Threshold Model-based approximation using direct input of data. It is important to note, however, that only four of the thirty predictions (4/30 = 13.3%) have a prediction error of greater than 0.006. In addition, all of the mean prediction errors are within 0.005. Given the multitude of factors that affect the ORIT and the randomness inherent to all biological action, the low error values provide supporting evidence for the accuracy of the RPORITA.

The most striking prediction errors occur on 29 March in the 2006 Fiji measles outbreak, the day of the most extreme error value of −0.0088 for the prediction with a PDD of 6. At this point, the |prediction error| mean is 0.0074, a much greater value than any of the other means. This extreme nature may be attributed to the relatively low DSI. This relationship is most likely caused by the high infectiousness, and therefore high variability, of the disease dynamics at such an early point in the ORI. Based on this fact, it appears that the RPORITA is best applied with a DSI of at least 10 days.

Based on **Tables 3** **and** **4**, the most accurate method for applying the RPORITA may be determined. An overarching trend cannot be established between either 1) the PDD and prediction error, or 2) DSI and prediction error. However, in both outbreaks, the prediction error mean is the highest when six days separate the day of data input and the day for prediction (PDD = 6). Overall, based on the numerical data presented in **Tables 3** **and** **4**, the two most accurate methods for applying the RPORITA may be established:

1. Predict the ORIT five days in advance (with overall mean |prediction error| of 0.00340). Or, more accurately,
2. Predict the ORIT four days in advance by averaging the predictions generated with PDDs of 4, 5, and 6 (with overall mean |prediction error| of 0.00223).

**Table 3:** Data demonstrating the two key relationships concerning RPORITA prediction error for the 2006 Fiji measles outbreak.

DSI	|Prediction error| mean	PDD	|Prediction error| mean
9	0.0074	4	0.00398
14	0.0021	5	0.00406
19	0.0013	6	0.00428
25	0.0042		
29	0.0055		

The prediction day difference (PDD) is the difference between the second day of direct input on which the prediction is based and the day of the prediction. The Days since Start of Immunization (DSI) is the number of days between the day of prediction and the start of the Outbreak Response Immunization. This data presents a numerical depiction of the two critical relationships with regard to Recursive Prediction of the Outbreak Response Immunization Threshold Algorithm (RPORITA) error: 1) between DSI and prediction error, and 2) between PDD and prediction error.

**Table 4:** Data demonstrating the two key relationships concerning RPORITA prediction error for the 2003 RMI measles outbreak.

DSI	|Prediction error| mean	PDD	|Prediction error| mean
19	0.0027	4	0.00320
24	0.0052	5	0.00274
29	0.0023	6	0.00336
35	0.0032		
40	0.0021		

The prediction day difference (PDD) is the difference between the second day of direct input on which the prediction is based and the day of the prediction. The Days since Start of Immunization (DSI) is the number of days between the day of prediction and the start of the Outbreak Response Immunization. This data presents a numerical depiction of the two critical relationships with regard to the Recursive Prediction of the Outbreak Response Immunization Threshold Algorithm (RPORITA) error: 1) between DSI and prediction error, and 2) between PDD and prediction error.

## Discussion

In this study, I developed a recursive algorithm (the RPORITA) for predicting the vaccination coverage required to reduce the individual reproduction number to less than one. I then tested the RPORITA against data from two actual measles outbreaks. In addition, I developed a model to demonstrate how changes in vaccination coverage affect changes in the individual reproduction number.

### Strengths

The ability to predict the ORIT would allow an outbreak control agency to better coordinate a future immunization drive intended to stop the outbreak. Several methods for predicting the threshold are available, most of which involve time based functions for the individual reproduction number, a crucial aspect in the calculation of the threshold [10]. With respect to other approaches for analyzing the individual reproduction number and the ORIT, the RPORITA developed herein differs primarily in its fundamental nature. The RPORITA, in contrast with other time-based approaches, allows each outbreak to essentially define its own dynamics. The RPORITA bases the prediction of the threshold on the previous threshold values within the specific outbreak, allowing for a more widespread application.

Another possible method for predicting the ORIT through the Threshold Model would involve the prediction of each of the necessary variables: *S, I,* and *R*. However, this approach requires three predictions, while the RPORITA requires only one, thereby reducing the number of opportunities for error to affect the results. In addition, the RPORITA provides a simpler method for the prediction of the ORIT, involving only a single recursive definition that may be quickly applied with readily available survey data. The only data input requirement of the RPORITA, besides the survey data from two consecutive days, is the number of vaccinations that will occur on each day until the prediction, the value of which is under the control of the outbreak control agency.

The individual reproduction number and herd immunity threshold have a complex relationship [10]. Perhaps the most basic distinction is that the individual reproduction number is a largely abstracted and theoretical value intended more to inform policy (whether or not certain outbreak control strategies are effective) than to quantify the amount of resources needed for immunization programs [15]. To determine the ORIT, the vaccination coverage that results in an individual reproduction number of less than one must be solved for [9], involving intermediary steps. In contrast, the predicted value for the ORIT generated using the RPORITA may be immediately applied to ORI without any of these interceding steps. Therefore, the direct prediction of the ORIT sidesteps any additional predictions or mathematical methods required by the reproduction number prediction.

### Limitations

I applied the RPORITA to only two outbreaks due to the paucity of available data necessary for its implementation (specifically the day-by-day breakdown of rash onsets and immunizations). However, the RPORITA development is based solely on the dynamics of the 2003 RMI outbreak, given the assumption that the recursive nature of the algorithm would allow for its wide applicability. I then tested the RPORITA on both the data used for the development (the 2003 RMI outbreak) and new test data (the 2006 Fiji outbreak). Although this data is not generally collected in databases, it would be readily available in the field based on real time survey data during an outbreak. As more data becomes available, the RPORITA must be applied to several additional outbreaks, those of both measles and other VPDs, to obtain a greater understanding of its accuracy.

Another key aspect of the RPORITA is that equation (8) only applies when the slope of the ORIT curve is less than zero. However, during the significant majority of the ORI program, the ORIT curve has a negative slope. At a time for which the ORIT curve has a positive slope, the outbreak control agency would still be identifying and formulating a response to the outbreak. Therefore, it is highly unlikely that this factor would interfere with the successful application of the RPORITA.

Other limitations of the RPORITA result from the Threshold Model on which it is based. This model assumes homogenous mixing of the population and the mass action principle and does not take into account the exposed portion of the population [19]. All of these aspects limit its accuracy. In this respect, several aspects of the RPORITA may be improved. The RPORITA must be applied to several more outbreaks, especially those of other VPDs, before being deemed fully ready for field application. In addition, the incorporation of more variables into the RPORITA, such as vaccine efficacy, quarantine, school closings, and heterogeneity of the population, would improve its accuracy. However, the simultaneous difficulty in determining these variables in real time for use in the RPORITA would limit their practical application.

Another limiting aspect involves the difficulty inherent to identifying those who could benefit from immunization, in other words: susceptible persons. For the RPORITA to accurately predict the ORIT, the vaccines must be used to immunize susceptible persons against the disease, although this limitation is by no means a fatal flaw of the RPORITA or the Threshold Model. All previously vaccinated persons and those who have presented or are presenting symptoms of the VPD may be legitimately excluded from the estimated susceptible pool for the purposes of the ORI. Those symptoms for measles include runny nose, red eyes, cough, small white spots, and a rash [7]. Once enough susceptible persons have been identified, the outbreak control agency may apply the RPORITA prediction by simply vaccinated the stated fraction of the population and ensuring, based on available data, that those vaccinated persons are susceptible.

### Conclusions

The immunization strategy discussed in this paper is not the only option for outbreak control agencies. In fact, there are three possible general courses of action with regard to ORI. The outbreak can run its course, maximizing the number of infections at the lowest cost. Or, the outbreak control agency can immunize as many persons as possible, thus minimizing the number of infections and maximizing cost. However, there is middle road, the one facilitated by the RPORITA developed in this research: the outbreak control agency can immunize the minimum number of persons required to achieve the ORIT at that point in the outbreak. This approach strikes a balance between these inversely related objectives by limiting both infections and cost, resulting in an optimal strategy for impoverished nations seeking to preserve limited funds.

It is duly noted that higher vaccination coverage will reduce the number of infections caused by the outbreak, as it would further reduce the individual reproduction number. However, once the individual reproduction number has become less than unity, the outbreak will eventually cease regardless of its exact value within the range from 0 to 1. The specific individual reproduction number determines the number of infections.

The model for the individual reproduction number in equation (19) can be applied to outbreak control strategy to determine the effects of vaccination on the ability of the VPD to spread through the population at different points in an outbreak. This equation incorporates three critical factors affecting the ability of vaccination to reduce the individual reproduction number: the point in the outbreak at which these vaccinations would occur (involves variables *c*, *S*, and *I*), the vaccination coverage before the new vaccinations (which determines *V*), and the number of additional vaccinations (). With this tool the time at which vaccination has the optimum impact on the individual reproduction number may be determined. Also, equation (19) may help answer the question: are these vaccinations worth their financial cost at this point in the outbreak?

Overall, the primary purpose of the RPORITA is to predict, several days in advance, the minimum number of vaccines required to achieve ORIT and thereby gradually stop an outbreak. This prediction capability would allow poorer nations to plan and coordinate an immunization drive that implements the minimum amount of resources needed to guarantee the end to a VPD outbreak at that point. Despite the moderate prediction error, considering the multitude of variables and factors that affect the ORIT during an outbreak, the RPORITA proves to be accurate in its prediction of the ORIT. Overall, the RPORITA strikes a delicate balance between real-time applicability (through simplicity) and accuracy, thus achieving the overall goal of this research.
